The article "A Correlation Analysis between SNPs and ROIs of Alzheimer's Disease Based on Deep Learning" was retracted in 2023. Reasons: signs of a paper mill; suspected computer-generated content; unreliable results or conclusions; lack of ethics approval or compliance.

# A Correlation Analysis between SNPs and ROIs of Alzheimer's Disease Based on Deep Learning

**DOI:** 10.1155/2021/8890513

**Published:** 2021-02-09

**Authors:** Juan Zhou, Linfeng Hu, Yu Jiang, Liyue Liu

**Affiliations:** School of Software, East China Jiaotong University, Nanchang 330013, China

## Abstract

*Motivation*. At present, the research methods for image genetics of Alzheimer's disease based on machine learning are mainly divided into three steps: the first step is to preprocess the original image and gene information into digital signals that are easy to calculate; the second step is feature selection aiming at eliminating redundant signals and obtain representative features; and the third step is to build a learning model and predict the unknown data with regression or bivariate correlation analysis. This type of method requires manual extraction of feature single-nucleotide polymorphisms (SNPs), and the extraction process relies on empirical knowledge to a certain extent, such as linkage imbalance and gene function information in a group sparse model, which puts forward certain requirements for applicable scenarios and application personnel. To solve the problems of insufficient biological significance and large errors in the previous methods of association analysis and disease diagnosis, this paper presents a method of correlation analysis and disease diagnosis between SNP and region of interest (ROI) based on a deep learning model. It is a data-driven method, which has no obvious feature selection process. *Results*. The deep learning method adopted in this paper has no obvious feature extraction process relying on prior knowledge and model assumptions. From the results of correlation analysis between SNP and ROI, this method is complementary to other regression model methods in application scenarios. In order to improve the disease diagnosis performance of deep learning, we use the deep learning model to integrate SNP characteristics and ROI characteristics. The SNP feature, ROI feature, and SNP-ROI joint feature were input into the deep learning model and trained by cross-validation technique. The experimental results show that the SNP-ROI joint feature describes the information of the samples from different angles, which makes the diagnosis accuracy higher.

## 1. Introduction

Alzheimer's disease (AD) is a disease of brain tissue defect, which is manifested by cognitive impairment, memory decline, comprehension, and judgment impairment or loss [1]. Mild cognitive impairment (MCI) is considered an early stage of AD. Without scientific intervention and treatment, early patients with AD or MCI will continue to deteriorate, seriously affecting their quality of life and the development of society. With the implementation of the Human Genome Project (HGP), in recent years, the interdisciplinary application of mathematics, computer science, and biology has formed Bioinformatics. It converts genes, proteins, and other biological molecules into digital signals and then uses information science methods to process and analyze the information [2–7], so as to understand the pathogenesis of diseases. The pathogenesis of AD is complex and may be related to many concomitant diseases, age, and other factors. Imaging genetics is the study of the relationship between brain image variation and genetic variation, to characterize the pathogenesis of gene variation on brain structure and function. SNP is a polymorphism at the DNA level, which is the key source of the occurrence and development of AD. Magnetic resonance imaging (MRI) technology has been proved to be an effective method for the detection of a variety of mental diseases such as AD. The candidate brain regions that may be related to AD are called ROIs by researchers. The density, volume, and other morphological characteristics of ROIs are applied to determine whether there are abnormalities in individual brain structure or function [8]. The analysis and mining of genetic and medical data to study the pathogenesis of AD can help to improve the early diagnosis rate of AD and provide support for the early detection and treatment of AD. At present, some methods of correlation analysis between SNP and brain ROI have been widely used to explore the pathogenesis and risk assessment of Alzheimer's disease [9, 10]. However, this strategy partially ignores the interrelationships between brain regions and may miss other important genetic variations that have not yet been reported.

In recent years, genome-wide association study (GWAS) has been applied to the study of different complex diseases globally [11, 12], and the relevant susceptible SNPs have been accurately identified and included in the GWAS Catalog [13]. With the generation of high-throughput whole-genome sequencing data, the role of data-driven genome-wide association research method on the pathogenesis of AD becomes more and more obvious [14–16]. However, with further research, it was found that the experimental results obtained by traditional GWAS are difficult to repeat, with low explanatory power and lack of heritability. Association analysis based on single variables can reveal some pathogenic loci or risk genes. For example, Westman et al. used the least square method to analyze MRI. In the experimental classification results, the accuracy of AD and normal controls was 87%, and that of MCI and normal controls was 71.8% [17]. Beheshti and Demirel calculated the Pearson correlation coefficient between the gray matter voxel features of MRI and the classification label, measured the correlation, and conducted feature ranking. By comparing different feature ranking methods, the final classification results of AD and normal controls were up to 88.8% [18, 19]. Most of the above studies are based on single-modal image data, but single-modal data usually only reflected part of the information related to brain abnormalities from a certain side, lacking statistical efficacy. The univariate association analysis ignored the weak markers, which produced significant changes by interacting with other molecules [20]. Multimodal neuroimaging data can provide complementary information and theoretically improve the accuracy of classification results. In order to systematically understand the formation mechanism of AD, multiscale, multimode, and heterogeneous data should be fused to mine the interaction between cross-omics variables [21, 22]. Some methods of data fusion based on ensemble classifier, dimension-based, and multicore learning have been proposed to establish a fusion predictor for other complex diseases. In addition, some studies have proposed improvement methods from the aspects of statistical learning [23] and regulatory relationship between SNP and gene [24].

With the development of computing hardware and the growth of data scale, the deep learning model [25] has been widely used in many application fields; for example, it has made remarkable achievements in biological and medical information processing, such as disease diagnosis [26–28]. So far, some risk genes that are significantly associated with AD have been excavated from the genomic level, but this may still be just the tip of the iceberg behind their complex genetic mechanisms. The complex interaction mechanism among genetic factors makes it difficult to understand the formation mechanism of AD, while the deep learning model has certain advantages for understanding nonlinear mapping. For AD classification, Nanni et al. first processed MRI features with different feature extraction methods to obtain multiple groups of features and then fused multiple groups of features with different combination methods to compare the differences of results generated by different methods [29]. Liu et al. used multimodal image data and deep learning network to extract depth features to achieve AD diagnosis, revealing the close relationship between changes in gray matter and AD disease [30]. Altaf et al. used Support Vector Machine (SVM), random forest, and *K*-Nearest Neighbor (KNN) to classify Alzheimer's disease and assigned a weight to each classifier. Finally, the classification results of each classifier were integrated and weighted [31]. Suk et al. proposed a method based on deep learning to distinguish NC (normal control) from AD, NC from MCI, and MCI from AD. However, the classification results are relatively insensitive to MCI [32].

In order to overcome the shortcomings of methods proposed by the previous researchers, we utilize a new strategy from the perspectives of feature fusion and automatic feature extraction. In this paper, we propose an analysis and diagnosis method of correlation between SNPs and ROIs based on deep learning. The method includes the following: on the hand of correlation of SNPs and ROIs, since deep learning model does not need to extract features manually, our method directly uses SNP data as input and uses the predicted value of ROIs as output to train the model; on the hand of diagnosis, first feature confusion is used on SNP data and ROI data, then a random forest algorithm is adopted for feature importance ranking, and finally a deep learning network is used to improve the performance of classification of disease state. Experimental results show that the error of our method is lower than that of other correlation analysis and diagnosis methods.

## 2. Methods

The study of the association between SNPs in the whole genome and ROIs in the brain region and predicting the patient's disease state is beneficial for early diagnosis and treatment of AD patients, but the current analysis and diagnosis method of the patient's disease state is almost always based on single-modal data, and the method may ignore the benefits of complementary information between SNPs and ROIs. In this paper, an analysis and diagnosis method of correlation between SNPs and ROIs based on deep learning is proposed, as shown in Figure 1, which is divided into three modules. Firstly, the SNPs and ROIs are confused with no feature information lost as much as possible. Then the random forest algorithm is used for feature selection. Finally, a deep learning network is constructed to predict the patient's disease state.

### 2.1. Random Forest Algorithm

Random forest (RF) is a popular ensemble machine learning method that has great application in both classification and regression tasks. Random is reflected in two aspects: the randomness of the sample and the randomness of the features. The implementation steps are as follows: firstly, the decision tree is constructed by randomly extracting part of the training set from the dataset through bootstrap technology; secondly, during the construction of the decision tree, features are randomly selected from the training set for splitting the nodes to ensure that they are the best partition. In the process of node splitting, there are usually Gini coefficient, information gain and information gain ratio to measure the goodness or badness of the partition.

RF uses only 66% of the original data to construct the decision tree. There is still about 1/3 of the data unutilized, which could be used to evaluate the performance of the decision tree and calculate the prediction error rate of the model, called out-of-bag data error. For each decision tree, select the corresponding out-of-bag data (out-of-bag (OOB)) to calculate the out-of-bag data error, noted as errOOB1. Randomly add noise interference to feature *X* of all samples of out-of-bag data OOB, and again calculate the out-of-bag data error, noted as errOOB2. Suppose there are *N* trees in the forests, then the importance of feature *X* = (∑errOOB2 − errOOB1)/*N*. The reason why this value can illustrate the importance of the feature is that, if after adding random noise, the out-of-bag data accuracy drops significantly (that is to say, errOOB2 goes up), it means that this feature has a great impact on the prediction results of the sample. This in turn indicates a higher level of importance. On the basis of feature importance, calculate the importance of each feature, and rank them in descending order for feature selection.

### 2.2. Deep Learning Classification Model

With the rise of deep learning, it is now widely used in the medical field. The main manifestation is the diagnosis of diseases with the help of medical images, including the classification of diseases and the localization of lesion, early diagnosis of diseases, and screening. Deep learning originates from artificial neural networks, which are composed of multiple single-layer and nonlinear networks superimposed on each other; Deep Neural Network (DNN) relies on the relationship between layers, and each layer is a higher level of abstraction of the previous layer, which can train huge amounts of data and has the ability to learn the essential features of a dataset. Compared to traditional machine learning, deep learning has two major advantages: one is the data-driven automatic learning of features, when there are a large number of features, reducing the subjectivity and time of manual feature selection, and the second is that the model deeper than shallow models has a hierarchical structure of nonlinear features, thus contributing to better modeling of very complex data patterns. In recent years, it has also received increasing attention in the classification of medical images and disease prediction. Lu et al. [33] proposed a new framework based on deep learning, which used multimodal, multiscale deep neural network to diagnose individual AD. This method had an accuracy rate of 82.4% in identifying individuals with MCI, achieved a sensitivity of 94.23% in classifying individuals clinically diagnosed as AD, and had a specificity of 86.3% in nondementia control group. To address the situation where the multimodal data are not all complete, Thung et al. [34] proposed a multitasking deep learning model. Complete MRI data, incomplete PET data, and multimodal data such as demographic information (i.e., age, gender, and education level) and genetic information were used as inputs, and then the subnet weights were updated based on the availability of each modal data section. The results showed that the method was superior to LRMC [35] and iMSF [36] and could be extended to complex imaging data. The main types of deep learning are top-down supervised learning, such as Deep Convolutional Neural Network (DCNN) and bottom-up unsupervised learning, such as Stacked Auto Encoder (SAE). Both types of learning models can be used to classify patient disease states. In this paper, we use the former.

In this paper, consider the large number of applications of deep learning networks in related fields; we build a three-layer convolutional neural network, which is divided into an input layer, an implicit layer, and an output layer. It consists mainly of convolutional layers, pooling layers, and a fully connected layer. The role of the convolutional layer is local perception, which perceives each local feature firstly and then performs a higher level of local synthesis to obtain global information. The excitation layer is a nonlinear mapping of the output of the convolutional layer. The pooling layer is mainly used for feature downscaling, compressing the number of data and parameters, reducing overfitting, while improving the fault tolerance of the model. The fully connected layer is used to get the final output through the Softmax function. It learns features from the sample effectively and avoids complex feature extraction processes. We use the Relu activation function for the first two layers because it iterates quickly and improves its generalization ability through the drop layer, and the last layer implements the classification of patient states through Softmax activation function. Finally, we evaluated the performance of the entire model, as well as a comparative analysis against models that did not perform biometric combinations.

Compared with traditional neural network activation functions, such as Sigmoid and Tanh functions, Relu function has following advantages: bionic principle makes it excellent for feature filtering, avoiding gradient explosion and gradient loss problems and simplifying the calculation process. Therefore, the Relu function is used as the activation function in this paper, and its definition is shown in

(1) $$\begin{array}{c} f\left(x\right)=\left\{\begin{array}{c} 0,\;\text{for }x<0,\\ x,\;\text{for }x\geq 0. \end{array}\right. \end{array}$$

Softmax is used in the process of multiclassification by taking the output of multiple neurons and mapping it to the (0,1) interval, which can be understood as probability, to perform multiclassification. The sum of probabilities for all classes is 1, and the class with the highest probability is selected as the classification result. The Softmax function is used as the activation function of the fully connected layer in this paper and for the probability that the sample vector *X* belongs to the *j*^th^ classification calculated as

(2) $$\begin{array}{c} P\left(y=j\right)=\frac{e^{x^{T}}Wj}{\sum_{k=1}^{K}e^{x^{T}Wk}}. \end{array}$$

## 3. Experimental Data and Evaluation Measures

### 3.1. ADNI Datasets

The neuroimaging program of Alzheimer's disease is the most influential of the current AD studies. ADNI (Alzheimer's Disease Neuroimaging Initiative) database (http://adni.loni.usc.edu/) is internationally one of the most widely used sources of experimental data. This study has full permission for using the dataset. The ADNI collected multimodal data such as images (MRI and PET, Positron Emission Computed Tomography), biological sample data (genetic data, cognitive tests, and blood biomarkers), and clinical statistics. MRI image data mainly reflect the changes of brain structure, including original data and preprocessed image files. PET imaging data reflect metabolic activity. Biological sample data include blood, urine, and cerebrospinal fluid (CSF), while clinical statistics consist of clinical information on each subject, including demographic, physical, and cognitive assessment data. The genetic data were sequenced by high-throughput sequencing data, and the sequencing file format provided by ANDI was VCF (Variant Call Format), BAM (Binary Alignment Map), etc. Studies have shown that genetic factors play an important role in AD. ADNI integrates genetic, imaging, and clinical data into a data platform for analysis, so as to facilitate global researchers to further study the occurrence and development mechanism of AD.

### 3.2. Experimental Data Preprocessing

The dataset used in this paper contains 632 samples, each of which has 486 SNPs and 56 ROIs. The evaluation index mainly adopts RSME (Root Mean Squared Error) and so on. Through analysis, it is found that there is a big difference between SNP and ROI data and there is a big difference in the value and range of result data among different ROIs in ROI data (for example, some ROIs are between -1000 and -100, while others are between 100 and 1000). Therefore, it is necessary to carry out normalization preprocessing to keep the data in the same range. The normalization preprocessing not only speeds up iterative convergence but also improves the accuracy. These advantages will be explained in the experimental results of correlation analysis.

Then, in this study, SNP data and ROI data were used as input to construct a classification model to predict the disease status of the samples (CN, MCI, and AD).

(3) $$\begin{array}{c} \left[\underset{X_{n*p}}{\underbrace{\begin{array}{cccc} s_{11} & \cdots & \cdots & s_{1p}\\ s_{21} & & & \vdots \\ \vdots & & & \vdots \\ s_{n1} & \cdots & \cdots & s_{np} \end{array}}}\underset{R_{n*q}}{\underbrace{\begin{array}{ccc} r_{11} & \cdots & r_{1q}\\ \vdots & & \vdots \\ \vdots & & \vdots \\ r_{n1} & \cdots & r_{nq} \end{array}}}\underset{Y_{n*1}}{\underbrace{\begin{array}{c} y_{1}\\ \vdots \\ \vdots \\ y_{n} \end{array}}}\right], \end{array}$$

(4) $$\begin{array}{c} \min\overset{n}{\underset{i=1}{\sum }}L\left(y_{i},f\left(S\right)\right) \end{array}$$

(5) $$\begin{array}{c} s.t.\min\left|S\right|, \end{array}$$

where *X*_*n*∗*p*_ matrix represents the SNP site value, where *n* represents the number of samples, *p* represents the number of SNPs, *S*_*ij*_ ∈ {0, 1, 2}, “0” represents the wild homozygous type, “1” represents the heterozygous type, and “2” represents the mutant homozygous type; *R*_*n*∗*q*_ represents the ROI matrix, where *n* represents the number of samples, *q* represents the number of ROI, and its value is a continuous real number; and *Y*_*n*∗1_ represents the label column of the sample. Equation (3) indicates that the task of multiclassification is to find a minimum SNP and ROI set *S*, and the accuracy of sample classification is the highest, in which *L* function is 0-1 loss function. The dataset adopted in this paper contains 632 samples, each of which has 486 SNPs and 56 ROIs, so there are 542 features. In order to improve the training efficiency of deep learning, the sample label coding method shown in Table 1 is adopted in this paper.

### 3.3. The Evaluation Index

The Receiver Operating Characteristic (ROC) curve has two main functions: (1) model selection—the best signal detection model, discard the second-best model; and (2) parameter setting—set the optimal threshold in the same model. In order to evaluate the performance of our method, the ROC curve is used to demonstrate the multiclassification performance of deep learning. The horizontal and vertical axes of ROC curve are FPR (false positive rate) and TPR (true positive rate), respectively.

(6) $$\begin{array}{c} \text{TPR}=\frac{\text{TP}}{\text{TP}+\text{FN}},\\ \text{FPR}=\frac{\text{FP}}{\text{FP}+\text{TN}}. \end{array}$$

TP represents true positive, FN represents false negative, FP represents false positive, and TN represents true negative.

In the process of model training, 5-fold cross-validation method is adopted; that is, 80% subset samples in the data set are randomly selected as the training data, and the remaining 20% subset samples are used as the test data.

## 4. Experimental Results

### 4.1. Correlation Analysis Results of SNP and ROI Based on Deep Learning

#### 4.1.1. Comparison of Normalized Pretreatment Results

To demonstrate the superiority of the proposed method, the deep learning method is compared with the three-stage method and group sparse model. Figures 2 and 3, respectively, show the ROI prediction results of various prediction models on RMSE indexes before and after data preprocessing. It can be found that the method is very similar in performance, but the method in this paper has no artificial feature extraction process.

Next, the normalization method is used to preprocess ROI data, and the results are shown in Figure 3. It can be found that the normalized pretreatment is beneficial to improve the efficiency of the regression method. The RMSE of the various methods decreases by several orders of magnitude, which also demonstrates the improvement of the model error by normalizing the data, further confirming the necessity of normalizing the ROI data, which has a very different and wide range of values stated in the analysis phase. The previous six methods are proposed by previous researchers, while the last two are BP (Backward Propagation) neural network methods that we proposed on the basis of deep learning grouped by gene and hierarchical clustering. The final results also showed that our BP neural network method based on deep learning retains its superiority over other methods.

Figures 4 and 5, respectively, show the MAE results before and after data pretreatment. The performance of all regression analysis methods has been improved after pretreatment, among which the ridge regression method is more significant.

Comparing our method with the remaining competing methods, we find that the BP method demonstrates an advantage in predicting ROI phenotypes on both RMSE and MAE evaluation metrics, as evidenced by smaller regression errors.

#### 4.1.2. Correlation Analysis between SNPs and ROIs

Firstly, ridge regression was used as the primary selection for SNPs, and the importance degree of SNPs was ranked according to their regression coefficient. After that all SNPs were divided into 33 groups by using the gene grouping data, and then the three regression methods were used for each group, respectively. Their regression error results are shown in Figure 6.

It can be found from Figure 6 that the deep learning method is superior to other regression analysis methods in almost every group of data. According to the gene grouping data, the SNPs (SNP21, SNP92, SNP431, SNP328, and SNP9) of the top 5 weight coefficients were in groups 2, 10, 26, 24, and 2, respectively. Next, the Pearson correlation coefficients between these key SNPs (the first 3, SNP21, SNP92, and SNP431) and ROI are shown, respectively, as shown in

(7) $$\begin{array}{c} r=\frac{\sum_{i=1}^{n}\left(X_{i}-\bar{X}\right)\left(Y_{i}-\bar{Y}\right)}{\sqrt{\sum_{i=1}^{n}{\left(X_{i}-\bar{X}\right)}^{2}}\sqrt{\sum_{i=1}^{n}{\left(Y_{i}-\bar{Y}\right)}^{2}}}. \end{array}$$

The Pearson correlation coefficients of the above SNPs and ROIs are shown in Figures 7, 8 and 9, indicating that different SNPs are complementary to ROIs, and the same SNPs have a strong negative correlation with different ROIs, while others have a strong positive correlation. Of course, these data are statistics only, and the results depend in part on the sampling process.

### 4.2. Results of Disease Diagnosis Method Based on Deep Learning

To illustrate the advantages of multimodal data feature fusion, the multicategory performance is shown in the following three cases: prediction based on SNPs only, prediction based on ROIs, and SNP-ROI joint prediction.

#### 4.2.1. Prediction Based on SNPs

In order to improve the training efficiency of deep learning model, the random forest method [37] was first used to evaluate the correlation between each SNP and the sample classification state, and then the correlation degree was ranked. The results are shown in Figure 10.

Due to the large number of SNPs, it is plotted at an interval of 20, and the other SNPs are omitted. The higher the correlation degree, the higher the contribution of the SNP to the sample classification. In order to save training cost, Top *K* SNPs can be selected as the input of the deep learning classification model.

It can be found from Figure 11 that when feature weight is extracted from Top 10 SNPs, the effect is better than other feature combinations, and the AUC (Area Under Curve) area in the ROC (Receiver Operating Characteristic) curve is 0.6.

#### 4.2.2. Prediction Based on ROIs

As in the previous section, the random forest method is still used to examine the degree of correlation between a single ROI and the sample state, and all ROIs are sorted by the degree of correlation, as shown in Figure 12.

Because of the large number of ROIs, they are plotted at intervals of 2, with other ROIs omitted. Using the ROI weight ranking results generated by the random forest. Selected weight Top 5, 10, ..., 50 ROIs were used as input to the deep learning classifier model, and then 5-fold cross-validation was used for model training.

The experimental results in Figure 13 show that when the 10 ROIs in front of the weight are extracted as the feature input, the AUC area in the ROC curve reaches 0.77, and compared with Figure 10, the ROI feature is better than the SNP feature to describe the sample's disease state. This result is consistent with intuitive cognition, because ROI can directly describe the characteristics of the individual's disease, while SNP is genetic data, which is only a potential pathogenic factor for the sample's disease state.

#### 4.2.3. ROI-SNP Jointly Predicting

ROIs can directly reflect the structural characteristics of the brain, while SNPs reflect the genetic characteristics of the sample. The former is more direct with the sample state, while the latter is a potential pathogenic factor, showing certain complementarity. Therefore, this paper intends to combine the two characteristics. Considering the combination of SNPs and ROIs, a random forest was used to calculate all the weights of SNPs and ROIs for ranking. The ranking results are shown in Figure 14.

The results in the figure reflect the above view that ROI is more directly related to the sample state. Using the weight ranking results generated by the random forest. Weight in front of 10, 20, ..., 100 SNPs and ROIs were used as joint feature input to train the deep learning classifier model, and the results are shown in Figure 15.

It can be found from Figure 15 that when the feature extraction weight ranks the top 10 SNPs or ROIs, the AUC area in the ROC curve reaches 0.8, which is better than the classification performance of SNP-only and ROI-only. The experimental results show that the combination of characteristics of different types of data is beneficial to provide complementary information, so as to obtain better sample classification accuracy.

According to the above ROC analysis results, with the increase of the number of features, the multiclassification results of various classification models show a certain degree of decline, which may be due to two reasons: (1) there is information redundancy, or even noise, between the features added later and the features added earlier, resulting in performance degradation; (2) due to the increase in the number of features, the deep learning classification model needs to consume more resources for training. If the training is insufficient, there may be underfitting of the model, resulting in performance degradation.

## 5. Conclusion

So far, some risk genes that are significantly associated with AD have been excavated from the genomic level, but this may still be just the tip of the iceberg behind their complex genetic mechanisms. Aiming at the problems of insufficient biological significance, large errors and inaccuracy of disease diagnosis in previous association analysis and disease diagnosis methods, we present a method of association analysis and disease diagnosis based on deep learning. Our method is a kind of data-driven method, which does not require prior knowledge to extract features manually, and the regression performance and multiclassification accuracy can also meet the application requirements. In addition, according to the experimental results of multiclassification tasks, the data fusion of complementary features is conducive to improving the accuracy of the model. In this paper, disease diagnosis can be regarded as a triad task. Each sample has three candidate states (normal, mild cognitive impairment, and AD). ROIs reflect the structural information of the brain, while SNPs reflect the genetic information of individuals, and the two information are complementary. In order to improve the disease diagnosis performance of deep learning, this paper uses the deep learning model to integrate SNP characteristics and ROI characteristics. On the experimental data set, SNP feature, ROI feature, and SNP-ROI joint feature are extracted, respectively, and these three features are input into the deep learning model, respectively, and trained by half fold cross-validation. The experimental results show that the SNP-ROI joint feature describes the information of the samples from different angles, which makes the diagnosis accuracy higher.

In this study, we proposed a correlation analysis of SNPs with ROIs and constructed a deep learning AD disease diagnostic model with SNP-ROI joint features. We uncovered a number of potentially pathogenic SNPs through correlation analysis and achieved an AUC of 80% with the SNP-ROI joint feature diagnostic model, as our model is data-driven and therefore does not rely on manually extracted features, which provides a clinical suggestion for existing AD diagnoses based on the physician's a priori judgement, and the improved diagnostic accuracy of the joint feature compared to a single feature, which gives us a research direction: firstly, the fusion of this genetic and imaging data for disease diagnosis is better than unimodal data; secondly, the physician's a priori information can be fused with other representative intermediate phenotypic features to further improve diagnostic quality.

Due to the limitation of computing resources, data, and data model, traditional image genetics research is mostly based on single mode image data. Since the single-modal brain imaging data only reflect some local information of brain structure or function, it is difficult to identify patients with early AD without obvious morphological changes. In addition, most of the studies used imaging genomics to investigate the genetic variation related to AD and only investigated the impact of genomic variation on AD. However, like other complex diseases, it is related to the interaction of multiple biomolecules. Only the analysis of omics data at a single level will make it difficult to explain the pathogenesis of AD. Therefore, we believe the following: (1) the multimodal brain image data packets contain more information than the single-modal image data packets, and the different modal image data have certain complementary information, so the establishment of multimodal brain image data fusion analysis model is conducive to the accurate identification of early AD patients; (2) on the basis of in-depth mining of genome-wide SNP data of AD, the integration of other levels of omics data is conducive to a systematic and complete understanding of the occurrence and development process of AD; (3) the construction of biomolecular interaction network and the identification of its key feature modules are conducive to improving the performance of MCI/AD classification or risk assessment models and can also help to explain the molecular mechanism of diseases from the perspective of network modules and biological pathways; and (4) based on the powerful computing advantages of cloud platform and feature extraction advantages of deep learning model, it is helpful to carry out deep mining of AD multimode image data and multisource omics big data.

## Figures and Tables

**Figure 1:** An analysis and diagnosis frame diagram.

**Figure 2:** The comparison results of RMSE on nonnormalized data.

**Figure 3:** The comparison results of RMSE on normalized data.

**Figure 4:** The comparison results of MAE (Mean Absolute Error) on nonnormalized data.

**Figure 5:** The comparison results of MAE on normalized data.

**Figure 6:** The regression results of feature group.

**Figure 7:** Correlation coefficient between SNP21 and all ROIs.

**Figure 8:** Correlation coefficient between SNP92 and all ROIs.

**Figure 9:** Correlation coefficient between SNP431 and all ROIs.

**Figure 10:** Correlation between SNP and sample label.

**Figure 11:** Multiclass classification results by SNPs.

**Figure 12:** Correlation between ROIs and sample label.

**Figure 13:** Multiclass classification results by ROIs.

**Figure 14:** Correlation between ROI, SNP, and sample label.

**Figure 15:** Multiclass classification results by ROI-SNP.

**Table 1:** Sample state coding diagram.

MCI	0	1	0
CN	1	0	0
AD	0	0	1

## Data Availability

Data are available at http://adni.loni.usc.edu/.
